# The Ergonomic Association between Shoulder, Neck/Head Disorders and Sedentary Activity: A Systematic Review

**DOI:** 10.1155/2022/5178333

**Published:** 2022-03-21

**Authors:** Rama Krishna Reddy Guduru, Aurelijus Domeika, Linas Obcarskas, Berta Ylaite

**Affiliations:** Institute of Mechatronics, Kaunas University of Technology, Kaunas, Lithuania

## Abstract

**Background:**

Work-associated upper limb and neck disorders are common occupational disorders throughout the world. These disorders are usually observed more in workers who spend a long time sitting, referred to as sedentary activity (SA). The immediate and distorted risk of sedentary-related problems was considered high in Europe, Australia, and the United States. Even though mediation is convenient, it is likely to reduce office workers' risks of developing cervical and upper body pain due to sedentary work. This systematic review addresses risk factors and evaluates the relationship between SA and upper body disorders in office workers (i.e., shoulder and neck/head).

**Methods:**

PubMed, Scopus, and Web of Science were searched for articles published between January 2010 and August 2021 in the English language. The three keywords “sedentary,” “upper body elements,” and “work” (and their derivatives) were searched to identify studies and carry out this systematic review. The articles were searched so that all three keywords or at least a derivation of each keyword should appear. *Findings*. Of the 40 articles that met the enclosure criteria, 32 studies examined the association of SA and upper body elements during both office and computer work. However, three articles were evaluated in the sit-stand work environment, and in the remaining five studies, one was evaluated during teaching, two during hospital work, and two during mixed working conditions.

**Conclusions:**

Research related to SA focuses mainly on extended risk factors, but there was no focus on other aspects, such as muscle and tendon contractions. As there is a convincing connection between SA and the upper body, our close examination identifies the need to institutionalize a system for collecting, analyzing, and describing the impact and short-term effects of SA on the upper body. Additionally, some suggestions were made to minimize the risk in a sedentary working environment.

## 1. Introduction

The lifestyle of people has changed vividly over the centuries. Initially, various work conditions were observed in the workplace, but today most people are stuck in the same place forever [1, 2]. Work-related musculoskeletal disorders (MSDs) are frequently connected with ergonomic risk factors such as contact stress and uncomfortable posture (changes in normal working posture). MSDs affect the neck, shoulders, and lower back (LB) and significantly impact a person's well-being and efficiency at work [3–5]. MSD associated with work is 70–80% in industrialized countries, indicating the need for treatment interventions [6, 7].

Upper body complaints have become more widespread among employees. Neck pain (NP) is quite prevalent and can cause physical exertion among office workers than other occupations [8, 9]. The annual frequency of NP in office employees ranges from 42% to 63%, with office workers having the highest incidence of neck problems (17% to 21%) among all other occupations. During a 1-year follow-up, around 34% to 49% of workers report a new beginning of NP [10–12, 12]. NP has a substantial effect on not just individuals but also on industry and society. Shoulder pain (SP) is the third most prevalent MSD among sedentary workers, with about 21% of all complaints. Rotator cuff disorders (RCD) such as bursitis, tendinitis, tendinosis, and degenerative tears are the most common causes. Rotator cuff tears, including tears of full and partial thickness, increase in prevalence over 40 years of age and are often asymptomatic; therefore, it may be appropriate to consider them as degenerative rotator cuff tears [4, 13–15]. In addition, an ongoing report indicates that office workers, especially those who work on personal computers, can also have a high risk of temporomandibular disorder (TMD) [16–19].

Few recent review articles examined the relationship between sedentary activity (SA) and health. Most of this information reported on the relationship between screen time and body composition but did not include other indicators of physical health (i.e., impact on the upper body). Furthermore, the studies on neck, shoulder, and hand problems among computer workers are unclear and difficult to understand. Many root causes of neck, shoulder, and hand problems, including physical exposure (i.e., motionless neck, arm posture, and performing repetitive and monotonous tasks) during work, are yet to be addressed.

As a result, to our knowledge, there are very few systematic reviews that address this particular issue focusing on the effects of SA on the upper body. So, the purpose of this systematic review is to distinguish the appropriate relationship between head, shoulder, and neck (HSN) disorders and SA and to evaluate the risk factors associated with SA, focusing on office workers.

## 2. Methods

### 2.1. Search Strategy

PRISMA was used to conduct the review and then to receive information from this systematic review [20]. The following databases were searched for relevant publications: PubMed, Web of Science, and Scopus. The three keywords “sedentary,” “upper body elements” (head, shoulder, and neck), and “work” (and their derivatives) were required to appear in the title or summary (Table 1). The following filters were applied: “English language,” “studies on humans of all ages,” “academic journals,” “between 2010 and 2021,” and keywords. Upon including the articles following the selection criteria, additional articles were identified by searching other sources.

### 2.2. Inclusion Criteria

The studies [cross-sectional (CSS) or cohort study (CS) and randomized clinical trials (RCTs)] were used if the following inclusion conditions were met: (1) a cohort of office staff without upper body pain was enrolled at the beginning of the study, (2) the essence of the job should be sedentary, (3) the onset of NSP was measured as a result, (4) reported an association between the physical risk of neck/shoulder due to SW, and (5) full-text articles available in English.

### 2.3. Exclusion Criteria

Conference proceedings, non-peer-reviewed papers, opinion papers, commentaries, case reports, abstracts, and systematic reviews were omitted from the study [21, 22]. Furthermore, studies were omitted if they were not addressing any physical activity or sedentary behavior.

### 2.4. Quality Assessment/Risk of Bias

The studies were assessed using a checklist developed by Rhodes et al. [2]. The tool was based on the Cochrane Collaboration's instrument for assessing the risk of bias. The tool comprised seven questions answered with yes (1) or no (0). A score of 6 to 7 indicates low bias and high quality; 4 to 5 indicate moderate bias and low quality; and 0 to 3 indicates severe bias and low quality [22, 23]. The assessment questions are as follows:

- Is there a theoretical framework in the study?
- Was an objective measure of SA used?
- Were the measures of SA reliable (e.g., pretested)?
- Was the study able to detect a nontrivial correlation?
- Was the study design an RCT?
- Was the baseline SA considered during the analyses (longitudinal analysis)?
- Was appropriate statistical analysis used?

#### 2.4.1. Data Extraction

A reviewer extracted the data, and the accuracy was validated by a second reviewer. Publication characteristics (author, year, study site), study demographics (age, sex, sample size), and evaluated risk factors were all retrieved from the eligible studies (Table 2). In addition, the type of work is distinguished (it must be more than half stable) [24–26]. Finally, the intervention, exploratory control, and various finalized estimates were noted.

## 3. Results

### 3.1. Search Results

The electronic database (i.e., Web of Science, Scopus, and PubMed) search yielded 2,680 articles, and 11 were identified from other sources (i.e., Google search). A total of 1425 articles were sorted after eliminating 791 irrelevant keywords and 475 duplicated articles, in which 1346 did not investigate the same case. Moreover, 17 that were systematic reviews, 16 that did not consider distinguishing between SA and physical inactivity, and six that did not contain humans were eliminated from the remaining 79 articles. Finally, 40 articles remained for the current review (Figure 1). Of the 40 articles included in this study, 27 were RCTs, eight were CSSs, four were CSs, and one was a quasi-experimental study (Table 2).

### 3.2. Methodological Quality Assessment

The quality assessment of the included studies is shown in Table 3. With 19 studies achieving a full score (7/7), the remaining 21 ranged between 4 and 6 [22]. The most typical deficiencies within the studies were as follows:

1. Fifteen did not pretest the SA reliability.
2. Eleven studies did not use baseline SA in the analysis.
3. Two studies did not achieve a nontrivial correlation.
4. Two did not use a statistically appropriate method for data analysis.

### 3.3. Assessment of SA

The article sought a clear definition and recognition of a sedentary lifestyle to confirm the disturbance between SA and physical inactivity. Of the 40 articles selected, 32 studies examined SA during office and computer work. Three articles assessed SA during a sit-stand work environment. The SA was assessed in the remaining five studies: one during teaching, two during hospital work, and two under mixed working conditions. SA of subjects in most of the studies are measured using questionnaires, visual observation, and videotaped, and apart from those, very few studies used accelerometers. Studies that estimated SA using questionnaires cannot conclude the proper estimation since the studies that used accelerometers showed an exclusive and objective estimation.

### 3.4. Assessment of Shoulder and Neck Disorders

Two articles examined SP, eleven studies investigated NP, and twelve examined shoulder- and neck-related disorders. The remaining studies only measured upper extremity disorders. Most of these studies used self-declared surveys to evaluate NSP, and the remaining studies used interviewing. In general, very few articles have focused on assessing neck/shoulder disorders using practical methods.

### 3.5. Evidence of an Association between SA and Neck Disorders

The majority of the employees work in an office setup, and almost all tasks are performed in a sedentary posture [4]. A desk, a chair, a computer (monitor, keyboard, and mouse), and sit-stand tables are included in the workstation. In this scenario, the association between SA and neck disorders was evaluated [10, 59].

Seven studies addressed the association between SA and neck disorders in the working population. In the working population, Kocur et al. found that forward head posture (FHP) had no significant influence on muscle stiffness, tone, and elasticity, nor did it increase the pressure sensitivity of superficial neck muscles in healthy, moderately symptomatic workers during the trial [32, 35, 60]. However, Petit et al. observed that intense physical work, awkward postures, substandard organizational ambiance, and age are risk factors for NP. The intrinsic risk factors of office workers often will have direct and indirect (intervene with the risk factors associated with the work environment) impact on the emergence of NP [8]. Moreover, Ehsani et al. revealed that long working hours in computers and prolonged sitting and standing were work-related factors that correlated with the occurrence of NP in office workers. Office workers with NP have a poor standard of living and constraints in performing their activities, for example, sleeping, indoor and outdoor activities, carrying heavy objects, doing social activities, and driving [39, 52, 61]. Overall, these findings demonstrate little evidence of the relationship between SA and NP in working populations. All reviewed studies highlighted the association and indicated the severity of work-related disorders in the neck.

### 3.6. Evidence of an Association between SA and Shoulder Disorders

Of the 10 studies, eight explored the effect of SA on shoulder disorders in the working population, while one study examined schoolchildren. Shariat et al.'s research focused solely on gender-based shoulder problems in the same workplace and found a positive correlation between pain severity in gender and both sides of the shoulder. The total pain score in the shoulders was revealed to be considerably associated with age [37]. According to Ng et al., the shoulder muscles contracted mildly to moderately during sedentary tasks. A significant difference in muscle activity was found in the head leaning and shoulder shrugging postures, but no demographic differences between male and female participants were found [3, 7, 55]. Zhu et al. researched the importance of positioning the forearm while typing and recommended that computer workers benefit by employing articulating armrests and frequent breaks. In circumstances where the forearm support cannot be placed at resting elbow height due to physical interference between workstation components or restricted desk adjustment, working in a floating arm posture may be preferable to working with forearms supported at an elevated height [53, 62]. In summary, there was conflicting evidence regarding the link between SA and shoulder problems in the working population due to discordant conclusions in various high-quality research.

## 4. Discussion

The findings of 40 studies on the association between SA and NSP were analyzed. Limited research and study heterogeneity showed little evidence of a link between SA and neck disorder in the working population, which led to these conclusions. In contrast, conflicting evidence was found for the association between SA and SP in the working population.

### 4.1. Summary of Main Results

People who work in the office are more likely to develop MSDs since they mainly include sedentary tasks for long periods. One example is the banking industry, where studies show that the prevalence of MSDs among bank employees ranges from 60% to 80%, indicating that they are particularly vulnerable to these injuries. The findings revealed that excessive periods of sitting among office workers could contribute to fatigue symptoms of MSD in various regions of the body, particularly in the upper extremities, neck, shoulders, and lower back. Fourteen studies (40% of all studies considered) showed that participants worked an average of 6.29 hours during an 8-hour work shift in a sitting position where females have been shown to sit longer than males (6.47 vs. 6.07 hours/day, respectively) [2, 37, 63]. For office workers, the prevalence of MSD in the shoulder and cervical spine has been reported to range from 40 to 80%. This high prevalence of MSD in workers may be due to uncomfortable and rigid postures and repeated motions in various parts of their bodies [57]. MSD is associated with both physical and mental aspects in office workers who spend significantly on computers.

Usually, due to a lack of time to engage in physical activity, office workers frequently suffer from MSD, particularly NSP. Some studies have shown that taking short breaks and walking during work reduces pain, and others reported that stretching exercises for 6–8 weeks pose benefits in reducing pain [53]. The basic principle underlying the benefits of stretching exercises, particularly for muscles, is that muscle tightness occurs due to a lack of physical activity [61, 64]. Previous research employed general flexibility exercises, but there was no evidence that these exercises reduce NSP in office workers. However, few studies have shown that thermotherapy and manual therapy can help reduce muscle soreness in office workers [31]. Still, there is currently no package of exercises designed specifically for flexibility and strength training for office workers.

#### 4.1.1. Assessment of SA

Studies suggest that SA increases all causes of mortality; doubles the probability of coronary disease, diabetes, and obesity; and increases the risk of bowel cancer, high blood pressure, osteoporosis, lipid disorders, depression, and anxiety. About 60 to 85% of people in the world adopt sedentary lives, making it one of the most serious, yet unrecognized, public health challenges of our day. Almost two-thirds of children are projected to be inadequately involved, with significant consequences for their potential well-being. Sitting time and increased muscle tension at work are associated with pain in the HSN, leading to an unfavorable work environment. When the neck and shoulder muscles are “overstrained,” the effect may be a sore spine, numb arm, and cold hands due to decreased blood supply or a mixture of these [34].

#### 4.1.2. Association between SA and Neck Disorders

Studies were conducted to analyze the association of SA with neck disorders. Interestingly, it was observed that there was limited evidence. The most common factors that increase the risk of developing NP among office workers are working hours on the computer, prolonged sitting, and forward flexion posture during work [39].

Workers are more likely to engage in physical labor, adopt awkward working postures, and live a sedentary lifestyle, whereas adolescents are less likely to engage in such activities. Paired with a sedentary lifestyle, adopting uncomfortable work postures for an extended period has been linked to NP. Therefore, increasing the level of physical activity among workers sought to prevent NP. Some studies evaluated the most common neck disorders and reported that computer workers with NP had a higher prevalence of TMD. Furthermore, the intensity of pain in response to cervical muscle palpation was significantly higher, and the pressure pain threshold of craniocervical was significantly lower among computer workers.

Additionally, this study emphasized the necessity of considering the work conditions of patients with TMD, as neck disability in computer workers is explained by the correlations between NP, TMD, and unfavorable work conditions [16, 35, 46]. Some studies suggest equipment such as a wearable sensor can help diagnose NP; participants had 8% lower neck flexion postures at sitting and standing workstations. Compared to the sitting workplace, the effect of the wearable sensor on the neck was more significant in the standing workstation [13, 65].

Many studies reported contradictory results on gender-specific effects on the neck among the working population. Women have a higher incidence of NP in the workplace than men, due to their diminutive stature and lower muscle strength. Furthermore, the “gender effect” on the results could be explained by different work activities (intensity, frequency, and type of exposure) [8]. Therefore, future studies could focus on a specific study population by considering the type of work and its impact on physical activity.

#### 4.1.3. Association between SA and Shoulder Disorders

The body of evidence regarding the relationship between SA and SP is more inconsistent than the relationship between NP and SA. In light of some studies, SP acquisition is undoubtedly due to working with arms above the shoulder level and other unbalanced positions, such as flexion of the front trunk, severe vibrations of the arm, pressing, and pulling the load. Moreover, other risk factors, such as physical discomfort situations, cuts, bending, working with arms raised to a support level, overloading, and handling heavy loads, can cause problems in the upper appendix, especially the shoulder problem [42, 55, 66]. In addition, computer and typography workers will generally work in a particular position. Unfortunately, working in a specific position with an unusual shoulder strap would put more weight on the shoulder and neck joints. Typically, SP, such as RCD, shoulder tendonitis, and NP affect sedentary workers.

The rotator cuff wears occur from repetitive behavior, putting tremendous strain on the rotator cuff tendons and the entire shoulder joint. Strains vary, from small, partial tears to massive, full, thick tears. Medical treatment for these tears would depend on the extent of the tear, the symptoms experienced by the injured worker, and the injured worker's age. Another type of workplace accident that occurs frequently is an abrupt traumatic injury, which can occur due to slipping and falling or being struck by a large object. Slips and falls frequently occur in the winter months or in warehouse-type facilities with cardboard, paper, and other packing items on the warehouse floor [47]. They usually occur when an arm is extended to break a fall or when the injured worker lands directly on the shoulder. When carefully adhered to, proper working positions can minimize the chance of maintaining an activity related to a rotator cuff sprain or tear [63, 67].

### 4.2. Explanatory Hypothesis of Divergent Results

Five factors are considered due to contradictory results in the study.

1. Duration of SA: this should be controlled according to the type of work.
2. Daily physical activity: regular SA may be enough to affect the upper body.
3. Testing time: the testing time affects the results for shorter and longer time activities.
4. Age of the participants: the relentless stable effects will be evident in more stable individuals than younger people.
5. A measure of SA: the measure may affect the stable measure of the results because emotional measurements (studies) cannot think much about measuring the time spent on SA.

### 4.3. Recommendations

This systematic review presented the absence of studies identified as probability factors due to the sedentary lifestyle in the upper body area. Mainly, the information showed contradictory results; it is speculated at various points to evaluate the effects on the HSN. This should be possible by analyzing more factors for extended periods or interventions for specific periods (days). These studies should suggest (1) specific surveys or measures that assess the reputation, regularity, and interval of SA and (2) specific questions or estimates of the completed physical training. Moreover, few technologies could be considered for detecting, analyzing, and restricting the SA. Ergonomic training is among them; it reduces the risk of MSD and the frequency of pain, even years after training [68]. Secondly, the usage of sensors is increasing in the work environment; the wearable sensor could be an effective tool to alleviate the postural stress of the head and neck in SW [31, 50, 65, 69]. Regarding detecting neck movements, the study of the wearable system by Lo et al. showed good performance in detecting repetitive movements [70].

## 5. Conclusions

The evidence from this review suggests the need to focus on appropriate work situations to manage their tasks efficiently by controlling the SA, rather than asking workers for regular exercise. Health outcomes (i.e., all-cause mortality, cardiovascular disease, MSD, diabetes, and depression) were consistently effective among workers. Therefore, it is necessary to control and prevent unnecessary SA. This can be initiated by preventive wellness projects, which can suggest work adjustments, such as signaling to urge workers to wake up every 20 minutes or recommend permanent work areas or dynamic workstations. Finally, more information on the outcomes of SA in physical well-being should be available to workers [51].

## Figures and Tables

**Figure 1:** PRISMA flowchart for systematic review.

**Table 1:** Search string used for study selection.

PubMed	Web of science	Scopus	Filters applied
(Title/Abstract (sedentary^∗^) AND title/Abstract (workers OR employees) AND title/Abstract (“upper body” OR shoulder OR head OR neck)	AB (sedentary ^∗^) AND AB (workers OR employees) AND AB (“upper body” OR shoulder OR head OR neck)	(TITLE-ABS (sedentary^∗^) AND (TITLE-ABS (workers OR employees) AND (TITLE-ABS (“upper body” OR shoulder OR head OR neck)	•The last 10 Years
			•English

**Table 2:** Characteristics of selected studies.

Study ID	Country	Year	Study design	N			Average age	Intervention	Subject Inclusion and Exclusion	Current status of follow-up	Work-Related Outcome
				Male	Female	T					
[27]	Japan	2021	RCT	57	18	75	20–59	Sit-stand desk	(i) Only desk workers were included.	Not active	The sit-stand desk effectively reduces SW and improves worker health and productivity.
									(ii) History of severe health complications was excluded.		
[10]	Taiwan	2021	QES	9	12	21	23.33 ± 2.9	Computer typing	(iii) Participants with no previous injury or surgery in the spine and abdominal regions were included.	Not active	Wearable biofeedback sensors may help computer users and sedentary workers to maintain a proper sitting position during their prolonged hours of desk work.
[2]	Iran	2021	CSS	105	149	254	37.12 ± 7.38	Office employees	(iv) Subjects with a history of previous illnesses were not included.	Not active	Among office employees, latent class-derived patterns can summarize MSD, and the chair's ergonomic design was strongly linked to the type of MSD patterns presented.

[28]	Switzerland	2020	RCT	-	-	120	18–65	Office work	(i) The severe health conditions of the neck were eliminated.	Not active	The expected outcomes are health-related productivity loss, neck disability, and pain.
									(ii) More than 25 work hours in a week in predominantly sedentary office work were included.		
									(iii) Participants who are expected to be in a long absence from work during the study period were eliminated.		

[29]	Brazil	2019	RCT	8	16	24	41.3	Sit-stand table	(i) Participants with self-reported MSD or low back, NSP, hand, or leg pain in the 3 months before the study were eliminated.	Not active	When 20–60% of the work was done standing rather than sitting, postural variability increased up to three times during computer work.
									(ii) Participants who self-declared computer usage for more than 4 hours during the work were included		
									(iii) Participants performing computer tasks for more than 5 years (the research aimed to study experienced workers performing tasks in the computer)		
									(iv) Absence from work for less than 1 month in the previous year, excluding holidays, was not considered.		

[30]	Iran	2019	RCT	30	15	45	34.62 ± 6.91	Sit-stand tables	(i) Participants with 1 year of working experience were included.	Not active	The time regime group positively affected energy expenditure, blood parameters, depression, fatigue, and productivity.
									(ii) There were several exclusions from the study, such as individuals who had underlying MSD or cardiovascular disease, those treated with psychiatric or hormonal control medicines, and those following specific diets or sports programs.		
[31]	Ethiopia	2019	CSS	318	436	754	42 ± 9.73	Teaching	(iii) Only teachers working at that institute were included.	Not active	Most survey members responded that they had SNP in the previous 12 months.

[32]	Poland	2019	RCT	-	-	50	25–55	Office workers	(i) Age between 25 and 55 years and BMI between 18.5 and 30 were recruited.	Not active	In healthy and mildly symptomatic office employees, FHP does not affect muscle stiffness, tone, or elasticity, nor does it alter the pressure sensitivity of superficial neck muscles.
									(ii) People with a weekly sedentary time of a minimum of 35 hours were included.		

[33]	Brazil	2019	RCT	-	-	69	49.3	Hospital workers	(i) An employee of the hospital and having a medical diagnosis was included.	Not active	This study found that most sedentary women take pain medication for MSD, indicating the need to improve workability.
									(ii) Referred to the rehabilitation center's physiotherapy service, women with at least one child were included.		

[34]	USA	2018	RCT	9	10	19	-	Computer work	(i) The participant with a typing speed of 30 words per minute was included.	Not active	Members with a portable sensor had flexible neck edges with 8% less and neck gravity with 14% less than members without a portable sensor.
									(ii) Subjects without pain in the upper body or region of the lower back within the past 7 days were included.		

[35]	Australia	2018	RCT	-	-	153	38.9 ± 8.0	Computer workers	(i) Participants who work at least 0.5 full-time equivalents were included.	Not active	There were no significant changes in pain; however, reducing longer sitting hours could reduce lower back pain. For more conclusive evidence, more samples and various interventions are required.
									(ii) Pregnant women were omitted.		
[36]	Egypt	2018	CSS	11	66	77	18–23	Sedentary office work	(i) Subjects with pain affecting the posterior or posterolateral aspect of the neck for more than 3 months were included.	Not active	NP individuals have reduced cervical lordosis and greater sternocleidomastoid compared to pain-free individuals.

[37]	Iran	2018	RCT	274	478	752	20–50	Office work	(i) Individuals with 1 year of experience in the present job were included.	Not active	The relationship between the intensity of pain at the shoulder level was examined.

[8]	France	2017	CSS	914	596	1510	30–49	Sedentary office work	(i) The participants mainly were blue-collar and low-level white-collar workers.	Still active	Musculoskeletal symptoms are observed after every follow-up stage, and work-related risk factors are identified.

[38]	Taiwan	2017	RCT	-	37	37	23–47	Hospital, factory, and university workers	(i) Participants without a history of accidents, traumatic injuries, or surgical treatment in the neck or upper limb regions were included.	Not active	It was revealed that aging might impact the mean blood flow in the shoulder region, causing it to increase discomfort. Paired with a sedentary routine and impaired microcirculation triggered by aging could evoke ischemia SP.

[39]	Iran	2017	CSS	-	-	220	24–60	Office work	(i) People with spinal deformities, history of neck surgery, malignancy, osteoporosis, neck tumor, multiple sclerosis, fracture or disorder of the neck region, trauma, and inflammatory conditions were excluded.	Not active	The incidence of NP was significant among office workers. Improving health conditions, reducing computer work hours, limiting extended sitting and static postures, having a break during work hours, and doing regular workouts were all flexible individual and work-related factors.

[40]	The Netherlands	2017	RCT	9	8	17	18–30	University students and staff	(i) Only university students and staff were recruited.	Not active	The results of the posture monitoring system after using a day demonstrated that it could help participants to improve their posture during their sedentary work.

[41]	Australia	2017	RCT	-	-	10	3–5	Computer work	(i) Participants' self-reported about their “diagnosed disorders” were excluded as it is likely to influence their participation in the study.	Not active	Children showed more significant mean head, trunk, and upper arm angles while playing with tablets than watching TV or playing with toys.

[42]	Sweden	2017	RCT	-	-	625	-	Cleaning, manufacturing	(i) Participants were excluded if they were predominantly white-collar workers.	Not active	Greater physical activity negatively affected the course of NSP.

[43]	Sweden	2016	CS	-	-	23794	18–65	Sedentary office work	(i) Participants with missing data on outcome or exposure were not included in the study	Not active	It is observed that leisure physical activity may reduce the risk of developing NP.
[16]	Brazil	2016	RCT	-	52	52	20–50	Computer work	(i) Any volunteer who had self-reported NP in the previous 2 years was excluded from the study.	Not active	The NP group has a higher level of disorders during computer-related work. The other group has no considerable effect.

[44]	Turkey	2016	RCT	-	-	116	-	Office work	(i) People who used computers for at least 10 hours and had no chronic disease related to the upper body regions were included.	Not active	The possibility of symptoms on the right side of the neck, wrist, and hand was fundamentally lower in the intervention group than in the reference gathering.
									(ii) Not being pregnant was another inclusion criterion for female participants.		

[45]	Turkey	2016	RCT	250	145	395	45.03 ± 8.85	Office work	(i) Individuals with chronic pain diagnosed with rheumatic disease and people who had received pain-related treatment within the last 3 months were excluded.	Not active	It is observed that MSDs are common in office workers and indicated the need for more attention to MSD and designing effective preventive interventions.

[46]	Portugal	2016	RCT	-	-	38	-	Office work	(i) Only sedentary workers with at least 1 year of experience were recruited.	Not active	Improvement in pain and increased adaptability were observed during work. The control group was observed to be more active, where few of them felt uncomfortable after long working periods.

[47]	Sweden	2016	CS	363	296	659	18–68	Office work	(i) Participants who self-reported blue-collar jobs as their primary occupation were included in the study.	Not active	Longer sitting hours can develop more pain severity in blue-collar workers over time.
									(ii) Participants who work in white-collar jobs, pregnancy, and adhesive allergy were excluded from the study.		

[14]	USA	2016	RCT	12	12	24	18–26	Computer work	(i) Participants who did not use the 10-digit touch typing method or did not experience MSD in the previous 3 months were excluded from the study.	Not active	Though sit-to-stand workstations may benefit health in the long term, there will be a trade-off for the musculoskeletal system, especially performing tasks in a sitting position during work.

[48]	Finland	2015	RCT	-	-	170	47.8 ± 10.8	Office work	(i) Subjects were included if they worked in an office the same way as other faculty members who worked in the original buildings with traditional seating workstations.	Not active	Most of the intervention subjects rated the sit-stand workstation's adjustability as good (83.3%), and 75.0% were satisfied with the workstation.
									(ii) Those who did not respond to the questionnaire were excluded.		

[49]	Ireland	2015	CSS	170	399	569	-	Office work	(i) Individuals who were employed for ≥1 year were included.	Not active	The study outcome shows significant differences in psychosocial exposure between age and sex, but no links were found between these differences and MSD symptoms.
									(ii) Subjects who had spent 50% or more of their day at the office and had spent at least 50% on computer work were only considered for further study.		

[50]	Thailand	2015	RCT	-	-	96	-	Office work	(i) Participants with a history of neck or shoulder surgery or abnormal neurological signs were excluded.	Not active	A regular exercise program that lasts about a month can reduce NSP. It also improves neck capacity and personal satisfaction for workers.

[33]	South Africa	2015	RCT	-	-	12	-	Sedentary typing work	(i) Subjects with spinal or neurological problems and a BMI of more than 25 or a high waist-hip ratio were excluded from the study.	Not active	When using a computer mouse, there are fewer postural dynamics at the cervical and thoracic spine locations than writing.

[52]	South Africa	2015	RCT	-	-	10	15–17	Computer work	(i) Subjects who (1) have a fully functional computer room; (2) offer CAT as a school subject; (3) have a similar computer laboratory setup were included in the study.	Not active	Head flexion is associated with upper quadrant musculoskeletal pain development for some time for a small group of students with significant 90 percent pain scores, balanced by age, sexual orientation, body mass index, computer use, and factors. Psychosocial.

[53]	France	2014	CSS	2161	1549	3710	38.7	Office work	(i) Each physician was requested to randomly choose 1 of 10 workers on the selected half-days of worker examinations.	Not active	The risk of neck disorders increased with a history of upper extremity MSD in men and decreased with BMI in women.

[54]	USA	2014	RCT	8	29	37	35.4	Office work	(i) Participants who worked at the facility for at least 1 year were included.	Not active	Specifically designed sit-stand tables or traditional table reminder software effectively introduced posture variability.
[55]	New Zealand	2014	RCT	8	9	17	20–26	Sedentary office work	(i) For this study, only right-handed participants over 18 and those who had not experienced any recent musculoskeletal pain were included.	Not active	The postures of head tilting and shoulder shrugging elicited significant muscular activity and showed no considerable changes in muscle activation between males and females.

[19]	Sweden	2014	CS	-	-	1153	30.5	Students	(i) Only students were included in the study.	Not active	The high prevalence of pain among nursing students and new graduate nurses indicates that prevention should be implemented early in nursing education. Still, they should also ideally be maintained postgraduation.

[56]	Norway	2012	CSS	8	19	27	18–65	Sedentary work	(i) At least 2 to 3 days per week of pain in the shoulder and neck area (unilateral or bilateral).	Not active	Pain levels fluctuate between “good” and “poor” days for subjects with low vs. high “central sensitization” indications than for the opposite.
									(ii) SW (mainly on a computer) and knowledge of Norwegian were also required.		

[53]	Korea	2012	RCT	12	12	24	25	Computer work	(i) Those who regularly use a computer in a seated position for more than 2 hours were included in the study.	Not active	Forearm assistance can help computer clients reduce physical anxiety when writing, only when their back is at the height of a resting attachment.

[57]	Canada	2012	RCT	2	13	15	36 ± 8.7	Computer work	(i) Participants with 2 and 23 years of experience (average 8.1) in computer-intensive sedentary environments were included.	Not active	Postural adjustments in the neck forward happened multiple times during each recording and differed considerably per participant, but not throughout the day.

[11]	Australia	2011	CS	759	724	1483	14.1	Computer work	(i) Only computer users were included in the study.	Not active	A multivariate model indicated that the probability of NSP increased in women. Computer use is related to NSP and posture in adolescents, but the association differs across boys and girls.

[58]	Republic of Korea	2011	RCT	20	-	20	23.6 ± 2.0	Sedentary work	(i) Workers who used the computer in a seated position during their work hours were included.	Not active	According to the findings, changes in activation patterns are associated with the cervical range of motion reductions, including flexion and lateral flexion.

C: control; N: study population; RCT: randomized control trail; CSS: cross-sectional study; CS: cohort study; QES: quasi-experimental study.

**Table 3:** Assessment of quality.

Study ID	1	2	3	4	5	6	7	Total score (7)
[27]	✓	✓	✓	✓	✓	✓	✓	7
[10]	✓	✓	✗	✓	✗	✓	✓	5
[2]	✓	✓	✓	✓	✓	✗	✓	6
[28]	✓	✓	✓	✗	✓	✗	✓	5
[29]	✓	✓	✓	✓	✓	✓	✓	7
[16]	✓	✓	✓	✓	✓	✗	✓	6
[31]	✓	✓	✗	✓	✓	✓	✓	6
[32]	✓	✓	✓	✓	✓	✓	✓	7
[33]	✓	✓	✗	✗	✓	✗	✓	4
[34]	✓	✓	✗	✓	✓	✗	✓	5
[35]	✓	✓	✓	✓	✓	✓	✓	7
[36]	✓	✓	✓	✓	✓	✓	✓	7
[37]	✓	✓	✗	✓	✓	✓	✓	6
[8]	✓	✓	✓	✓	✓	✓	✓	7
[38]	✓	✓	✓	✓	✓	✓	✓	7
[39]	✓	✓	✓	✓	✓	✓	✓	7
[40]	✓	✗	✓	✓	✓	✓	✗	5
[41]	✓	✓	✓	✓	✓	✓	✓	7
[42]	✓	✓	✗	✓	✓	✗	✓	5
[43]	✓	✓	✗	✓	✓	✓	✓	6
[16]	✓	✓	✓	✓	✓	✓	✓	7
[44]	✓	✓	✗	✓	✓	✓	✓	6
[45]	✓	✓	✓	✓	✓	✓	✓	7
[46]	✓	✓	✓	✓	✓	✓	✓	7
[47]	✓	✓	✓	✓	✓	✓	✓	7
[14]	✓	✓	✗	✓	✓	✗	✓	5
[48]	✓	✓	✓	✓	✓	✓	✓	7
[49]	✓	✓	✓	✓	✓	✓	✓	7
[50]	✓	✓	✓	✓	✓	✓	✓	7
[35]	✓	✓	✗	✓	✓	✗	✓	5
[52]	✓	✓	✓	✓	✓	✓	✓	7
[53]	✓	✓	✗	✓	✓	✓	✓	6
[54]	✓	✓	✓	✓	✓	✓	✓	7
[55]	✓	✓	✓	✓	✓	✓	✓	7
[19]	✓	✓	✗	✓	✓	✗	✓	5
[56]	✓	✗	✓	✓	✓	✓	✓	6
[53]	✓	✓	✗	✓	✓	✗	✓	5
[57]	✓	✓	✓	✓	✓	✓	✗	6
[11]	✓	✓	✗	✓	✓	✓	✓	6
[58]	✓	✓	✗	✓	✓	✗	✓	5

## Data Availability

The data generated and analyzed during the study are included.

## Abbreviations

SA: Sedentary activity
SW: Sedentary work
NP: Neck pain
SP: Shoulder pain
NSP: Neck and shoulder pain
HSN: Head, shoulder, and neck
FHP: Forward head posture
MSD: Musculoskeletal disorder
RCD: Rotator cuff disorders
TMD: Temporomandibular disorder
PRISMA: Preferred Reporting Items for Systematic reviews and Meta-Analyses
RCT: Randomized control trail
CSS: Cross-sectional study
CS: Cohort study.
BMI: Body mass index
